# The Artificial Intelligence and Neural Network in Teaching

**DOI:** 10.1155/2022/1778562

**Published:** 2022-06-10

**Authors:** Qun Luo, Jiliang Yang

**Affiliations:** ^1^Information Engineering Department, ChongQing City Vocational College, Yongchuan, ChongQing 402160, China; ^2^Henan Polytechnic Institute, Nanyang, Henan 473000, China

## Abstract

This study aims to explore the application of artificial intelligence (AI) and network technology in teaching. By studying the AI-based smart classroom teaching mode and the advantages and disadvantages of network teaching using network technology and taking the mathematics classroom as an example, this study makes an intelligent analysis of the questioning link of classroom teachers in the teaching process. For the questions raised by teachers, the network classification models of convolutional neural network (CNN) and long short-term memory (LSTM) are used to classify the questions according to the content and types of questions and carry out experimental verification. The results show that the overall performance of the CNN model is better than that of the LSTM model in the classification results of the teacher's question content dimension. CNN has higher accuracy, and the classification accuracy of essential knowledge points reaches 86.3%. LSTM is only 79.2%, and CNN improves by 8.96%. In the classification results of teacher question types, CNN has higher accuracy. The classification accuracy of the prompt question is the highest, reaching 87.82%. LSTM is only 83.2%, and CNN improves by 4.95%. CNN performs better in teacher question classification results.

## 1. Introduction

With the advent of the era of intelligence, schools and society are demanding to cultivate more innovative talents. This also puts forward new requirements for classroom teaching reform in the main links of education and teaching [1]. The development of information technology has led to the digitization of teaching. The disadvantages of the traditional teaching model are gradually highlighted. Combining the teaching of various disciplines and artificial intelligence (AI), big data, and various network technologies adopts new technical means to transform traditional classrooms into smart classrooms [2]. The smart classroom combines teaching content and information technology to make the boring classroom, which is originally the main output of teachers, vivid and interesting. Not only can students explore, cooperate, and communicate in an intelligent learning environment and give play to students' subjective initiative in learning, teachers can also communicate with students in real time through different teaching links. Teaching is no longer static but dynamic and variable. This not only facilitates the effective implementation of teaching tasks but also enables precise education and individualized instruction according to the teaching situation of different students, thereby improving the teaching effect [3–5].

AI has been widely used in higher education, providing technical support for practical teaching in universities and colleges. Yang et al. (2020) [6] studied the cultural industry management major of China Three Gorges University and created a practical teaching model based on AI. Firstly, they took massive open online courses and self-paced open courses to build an intelligent management cloud platform for practical teaching. Meanwhile, AI technology is used to realize personalized learning and provide intelligent push services. In this way, the online platform seamlessly integrates teaching content into specific teaching scenarios and uses the offline cloud platform to manage the teaching process intelligently. Tedre et al. (2021) [7] described how to teach the basics of AI to high school students who participated in interactive workshop activities. These activities take place in the context of a strategic plan to advance careers in science, technology, engineering, and mathematics. They include students learning how to build unbiased datasets, how to build interpretable classifiers, and how to build multimodal explanations. With the help of computer technology, AI teaching can quickly provide students with a virtual environment to experience the first-hand information of this process, helping them to understand better what they have learned [8].

Aiming at the shortcomings of the existing AI computer-aided design teaching system technology based on modern education theory and utilizing existing information, He and Sun (2021) [9] pointed out that AI computer-aided teaching has a system model teaching and collaborative learning functions. According to the development mode and application requirements of smartphones and AI computer-aided teaching, they proposed a teaching system model based on AI technology. In the process of theme logo design in a research study based on a digital network learning platform, AI computer-aided art teaching model has played an important role. Tiwari (2020) [10] introduced a convolutional neural network (CNN) model for fuzzy classification. The model classifies blur in gesture images into four blur categories: motion, defocus, Gaussian, and box blur. Chen (2021) [11] proposed an online oral English teaching platform based on the Internet of Things (IoT) to overcome the problems of low fluency and operability of the current online oral English teaching platform. The platform uses the IoT to design the architecture of the online spoken English teaching platform. A virtual teaching environment is constructed. A spoken English teaching system is used to correct the user's pronunciation and mouth movements. A part-of-speech tagging model based on long short-term memory (LSTM) is constructed. The attention mechanism is introduced in the LSTM network.

Methods of literature research and model validation are used to study the application of AI and CNN in smarter teaching. The innovation lies in the application of CNN and LSTM models in classifying questions in teaching classrooms, which is helpful for intelligent analysis of teachers' questions, thereby improving the teaching effect and realizing accurate teaching.

## 2. Materials and Methods

### 2.1. AI-Based Smart Classroom

AI provides powerful technical support for the intellectualization of distance education [12]. Students' thinking paths and their problem-solving potential target structures are tracked, and students' understanding domains are diagnosed and evaluated using expert systems, natural language processing, artificial neural networks, machine learning, and other technologies. These can provide students with timely guidance, feedback, and explanation. By analyzing the platform's big data, students' learning activities are planned with the appropriate level of difficulty and the most relevant content further to promote efficient learning behavior [13–15]. AI education has enriched the range of educational resources and made teaching methods more flexible. Teaching links and processes have been optimized. Meanwhile, in the teaching process, AI provides technical support for smart education, such as smart correction and case-based reasoning. These methods have injected fresh blood into education [4]. For example, machine marking reduces the burden on teachers. Teachers can have more time and energy to focus on student interaction, instructional design, professional development, and education quality. The AI-based teaching model is shown in Figure 1.

In Figure 1, the intelligent teaching system analyzes the teaching and learning status of teachers and students through the expert system, making the teaching process more intelligent and improving the teaching efficiency. AI is positioned as the forthcoming fourth technological revolution [16]. The revolutionary nature of AI is not only manifested in the advancement of technology itself, but it is more shocking than any previous technological revolution. It may even lead to changes in the relationship between people and technology [17]. The network makes the influence of distance on education fairness less and less. Filtering out the best explanations of a certain knowledge point by the best teachers from video resources has gradually reduced the necessity for many junior teachers in ordinary primary and secondary schools to teach conventional knowledge. AI's collection and optimization of this excellent video resource will enable it to undertake and be competent for regular teaching tasks. Traditional teaching concepts will be greatly challenged. The function of teachers will increasingly tend to play the role of “life mentor”. Teachers teach learning methods instead of knowledge points, guide students to learn independently, teach students the principles of life and behavior, and cultivate students' emotional intelligence, personality, and teamwork spirit. After AI frees up teachers' time, they will have more and more energy to pay attention to the individual development of each student.

The teaching process in the traditional classroom cannot be recorded and stored [18]. With the maturity of electronic schoolbags and interactive classroom technology, teachers use electronic equipment to teach and students to learn. They can use equipment to record knowledge points. This can become classroom process data for analysis. A complete teaching process dataset often encompasses classroom data, such as students' facial expressions, videos, and audio data. Through the statistical analysis model, the big data analysis model can realize the analysis of the teacher's teaching and the individualized learning analysis of each student. Intelligent homework correction is a typical application that uses big data technology to solve semantic recognition problems. At present, the similarity between the correction of English composition and the manual correction of excellent teachers has reached more than 95%. This shows that it can replace the heavy workload of teachers correcting English composition. The advantage of the machine is also reflected in its ability to allow students to modify it repeatedly. A typical human-computer collaboration teaching mode is shown in Figure 2.

Online teaching through online platforms and mobile platforms can expand the scope of everyone's learning and can also add more extracurricular knowledge. Meanwhile, online courses have advantages and disadvantages. The advantage is as follows: when students face the computer, it can prompt students to establish their dominant position in the learning process. Learning in the context of the network embodies true teaching following aptitude. Student learning is not limited by the age of entry and can avoid the time and space constraints in the traditional teaching model. The network environment is the liberation of time and space for students. A relaxed learning atmosphere can enable students to develop their talents. They can inspire each other, collaborate, communicate in learning activities, and learn to communicate and cooperate. Learning under the network background is a multidirectional information exchange activity. Students can compare, brainstorm, learn from each other, deeply understand, and digest the knowledge they have learned when they obtain different learning resources, which is beneficial to construct the meaning of new knowledge. However, some deficiencies still exist: for example, the online education realized through the Internet has significant regional differences in China. Affected by infrastructure construction, the developed areas in the east are better than the underdeveloped areas in the west in terms of the depth and breadth of online education. Therefore, the standard procedure for online education is objectively poor. There is a big difference between online education and traditional full-time education, mainly reflected in the asynchrony between teachers and students in time and space. A relatively single teaching mode has a tremendous negative impact on students' learning. It is mainly manifested in the decline of students' enthusiasm and initiative in learning and students' inaccurate grasp of the depth and breadth of teaching content, which affects the quality of teaching. Because the education and teaching process is realized through the network, teachers and students are not required to be strictly asynchronous in time and space, which objectively results in poor teaching interaction.

### 2.2. The Application of Network Technology in Teaching

The networked classroom based on network technology is a remote online interactive training classroom on the Internet. It usually uses network transmission technologies such as audio and video transmission and data collaboration. It can simulate the real classroom environment and provide students with an effective training environment through the network [19–21]. Firstly, students connect to online classroom applications or use a browser directly. Then, the account is logged in to the client provided by the online classroom administrator. Finally, students will participate in online teaching content in real time. The core of the online classroom is the sharing of teaching resources and collaborative browsing. Students can study anytime and anywhere without space restrictions. The new form of network teaching technology is shown in Figure 3.

In Figure 3, the new form of online teaching has significantly changed the status of teachers and students. The teacher's teaching process is networked and automated. Students' learning is more autonomous and diverse. They can conduct purposeful learning according to their own learning needs, which can improve their learning efficiency and increase their interest in learning. The key to the computer multimedia communication technology used in network technology teaching lies in the network communication protocol. According to the agreement, the communication computer compresses the sound, video, data, etc., and sends it to different places. The network receives compressed signals, such as voice, video, and data from different places, and the system control signal of the server. Decide which signals to decompress and display according to the requirements of system control signals. At present, the distance education system mainly relies on the Internet, computer, and multimedia communication technology, especially the latest streaming media technology from Real, Microsoft, and Apple, which can adapt to the network bandwidth. This enables students to see the real-time rebroadcast of teachers' lectures in remote classrooms in remote teaching classrooms and can get guidance from teachers, and teachers can also get feedback from students. The system usually uses Real-Time Transmission Protocol (RTP) [22], Real-Time Transmission Control Protocol (RTCP) [23], Real-Time Streaming Protocol (RTSP) [24] as real-time video and audio stream synchronization and flow control. This achieves data flow and broadband control and supports real-time broadcast and multichannel playback, as well as audio and video compression and decoding systems.

Although online teaching has many advantages, compared with offline learning at a fixed time and a fixed location, online teaching has fewer limitations to these environmental factors. Students only need to cooperate with the teacher's class time. Online education reduces commuting time, allowing students more time to review and preview. The learning effect of students will also be better. However, online learning also has higher network transmission requirements of hardware devices and server processing speed. With the increase in the number of people online simultaneously, the network will be stuck and delayed. These circumstances have certain requirements for students' self-control. Therefore, in teaching design, teachers can cooperate with real-time video, voice interaction, and other methods to give students a sense of offline learning.

### 2.3. Analysis of Teachers' Questions in Class Based on Deep Learning

AI technology is used in classroom teaching. This promotes the development of smart classrooms. Meanwhile, education and teaching also put forward new requirements and challenges to AI. Classroom questioning is an essential element in classroom teaching. AI is used to analyze classroom questions. Data-driven concepts are used to help teachers discover teaching patterns, for example, the dynamic relationship between the type of questions in the classroom and students' cognitive level. Machine learning algorithms are used to evaluate the learning effects of teachers' classroom questions. This not only facilitates the formation of teaching evaluation results but also analyzes the common problems of teachers' classroom questions. Teacher training is organized in a targeted manner, and personalized recommendation strategies are formulated.

For the analysis and research of teachers' classroom questions, most of them use video analysis. It not only requires a lot of labor and time costs but also requires manual coding, which is poor in portability. Although it can also analyze the law of classroom questions to a certain extent, it cannot be independently analyzed for large-scale videos, which is challenging to carry out. This demand promotes the emergence of intelligent analysis methods. AI-based natural language processing technology can reduce manual operations in classroom teaching analysis and has the advantages of accurate classification, real-time monitoring, and convenient large-scale expansion. Therefore, the proposed intelligent analysis method of deep learning is used to analyze and code classroom questions.

Questions in mathematics classrooms are regarded as research objects. The classroom questioning corpus is divided according to the content of the question and the type of question, combined with the characteristics of the corpus in daily classroom teaching and the cognitive level of students. The questioned content is divided into “0” which represents the type of basic knowledge points, “1” represents the type of topic information, and “2” represents the type of self-management. Types of knowledge points ask questions based on specific knowledge points to investigate students' mastery of basic knowledge, reasoning, and analysis abilities. The type of topic information is given by the teacher based on the topic's specific information. It tests students' understanding of specific topics, problem-solving ideas, reasoning, and other abilities. Self-management type of questions are questions for students' self-evaluation and self-reflection.

According to the question type, it is divided into “0” for the basic memorization type, “1” for the prompt type, “2” for the analysis type, “3” for the application type, and “5” for the evaluation type. The memorization type is a question the teacher asks to help students recall the knowledge they have learned. The prompt type is the teacher's prompt to the analysis process of a certain topic in the teaching process. Analytical questions are questions that teachers describe in terms of specific phenomena. Applied questioning refers to the teacher asking students to use the concepts they have learned and the knowledge they have mastered in the past to solve new problems jointly. Evaluation-type questions are questions that the teacher asks to summarize the students' knowledge.

Figure 4 is the specific operation flow of the designed mathematics classroom questioning classification based on deep learning. It is made of original data collection and organization, manual corpus labeling, data set preprocessing, vector representation and data sampling training, and final model evaluation. The original data collection uses 60 sessions of excellent model classroom records of junior middle school mathematics in the open data platform. The video is converted into text, and the teacher's question is extracted to form a data set. Then, they are labeled according to the content and type of the question. The questioned content is marked as “0”, “1”, and “2” according to the classification. The types of questions asked are marked as “0”, “1”, “2”, “3”, and “4” according to their classification.

The sorted data set is preprocessed. On the one hand, question sentences that are too long or too short, or the transcription process is wrong and ambiguous. This can reduce the noise in the corpus. On the other hand, the order of the corpus is shuffled before inputting the program, and the model construction is the result of the disorder learning. The content of the teacher's classroom questioning is often the question of the topic information type, and the other two are less. The mixed sampling method is used in the sampling process of sample collection. In order to prevent unbalanced datasets caused by misclassification, arbitrarily increase the number of corpora and collect data for a small number of question types, and reduce the corpus data collection for many question types, the same problem exists in the question type dimension. A suitable corpus classifier has a greater impact on the final classification result. The CNN model has advantages in text feature extraction, and LSTM can well retain the contextual semantic information in the text sequence. Therefore, CNN and LSTM are used as classification models for teaching classroom questions.

A CNN is a deep learning model or multilayer perceptron like an artificial neural network commonly used to analyze and process visual data. CNN is inspired by a biological process in which the pattern of connections between neurons is very similar to the organization of the animal visual cortex. Each cortical neuron responds to stimuli only within a limited area of the visual field. The receptive fields of different neurons partially overlap to cover the entire field of view. It consists of the data input layer, convolution calculation layer, ReLU excitation layer, pooling layer, and fully connected layer. The composition of the network structure is shown in Figure 5.

In Figure 5, CNN is used in various fields. For example, image segmentation, object segmentation, style transfer, etc., are all based on the feature extraction of images by CNN. The input layer of CNN is mostly *n* × *m* × 3 RGB images, i.e., red, green, and blue. In a convolutional layer, the input weight matrix for a region is called a filter. The filter slides over the entire image, repeating the same dot product calculation operation. The number of channels in the filter must match the number of channels in the input image. Typically, as the network goes deeper, more filters are used. The principle is that using more filters means more edge and feature detection. The two most used pooling methods are average pooling and max pooling. The latter is used more often. In CNN, pooling layers are used to reduce the spatial dimension but not the depth of the network. When using the max-pooling layer, the most sensitive region features points in the image in the input region of the *n* × *m* matrix is taken, and when using the average pooling layer, the average feature points of the input region are taken.

LSTM is the most used recurrent neural network. It solves the gradient explosion and gradient disappearance of the recurrent neural networks and can learn long-term dependence. Time series forecasting is widely used. It has more “doors” concept than other types of neural networks. In digital circuits, circuits with complex functions are formed through an organic combination of “AND gates”, “OR gates”, and “Exclusive-OR gate”. The three gates select information through the activation function and send it to the memory cell. The memory cells update the historical information of the state parameters. It can combine historical information for current tasks. For example, it can use the information contained in the frame of the previous video file to help understand the current image frame or predict the words that may appear later based on the text information before the sentence. The network structure is shown in Figure 6.

Part of the original data is deleted to ensure the balance of the collected classroom questioning corpus. Each type of data selected collectively is classified according to 6 : 2 : 2. The data is divided into a training set, validation set, and test set. The training set is used to train the original model. The validation set is used to adjust the parameters. It adjusts the parameters of the original formed model and optimizes the original model. The test set is used to test the absolute accuracy of the model. The distribution of various corpora is shown in Table 1.

In Figure 6, some original data have been deleted to ensure the balance of the classroom questioning corpus collected. Then, each type of data selected in the dataset is classified according to 6 : 2 : 2. The data is divided into the training set, validation set, and test set. The training set is used to train the most primitive model, and the validation set is used to adjust the parameters. That is, it is used to adjust the parameters of the original formed model to achieve the purpose of optimizing the original model. The test set is used to test the absolute accuracy of the model. The distribution of various corpora is shown in Table 1.

The classification result evaluation of class question classification uses accuracy, precision, recall, and F1 values as evaluation indicators. Accuracy represents the proportion of correctly predicted results to the total sample size. Precision is the probability that all predicted positive samples are positive samples. The recall is for the original sample, representing the probability of being predicted to be a positive sample among the actual positive samples. The F1 score considers both the precision rate and the recall rate so that both can reach the highest level at the same time and achieve a balance, that is, a comprehensive evaluation of the performance of the classifier. The specific calculation is shown in equations (1)–(4):

(1) $$\begin{array}{c} \text{Accuracy}=\frac{\text{TP}+\text{TN}}{\text{TP}+\text{FP}+\text{TN}+\text{FN}}, \end{array}$$

(2) $$\begin{array}{c} \text{Precision}=\frac{\text{TP}}{\text{TP}+\text{FP}}, \end{array}$$

(3) $$\begin{array}{c} \text{Recall}=\frac{\text{TP}}{\text{TP}+\text{FN}}, \end{array}$$

(4) $$\begin{array}{c} \text{F}1=\frac{2*\text{Precision}*\text{Recall}}{\text{Precision}+\text{Recall}}. \end{array}$$

TP represents the number of positive samples that the classification model predicts correctly. FP represents the number of positive samples that the classification model predicts incorrectly. TN stands for the number of negative samples that the classification model predicts correctly. FN represents the number of negative samples that the classification model predicts incorrectly.

The simulation experiment environment adopts Intel(R) Core (TM) i7-9700K CPU, memory is 64 GB, and the operating system is 64-bit Windows 10. The CNN and LSTM models are built based on the Keras framework [25], the number of iterations is set to 100, the batch size is set to 64, and the random deactivation ratio is set to 0.2. “learning_rate” is set to 1e-3. The number of convolution kernels in the CNN model is 256 and 5. A global max-pooling operation is employed. The number of neurons in the fully connected layer is set to 128. The Softmax function is used to classify the question texts in teaching classrooms. LSTM uses 128 hidden layer neural units to learn semantic information, connects two hidden layers into the fully connected layer, and uses the Adam method [26] to optimize the algorithm. The Softmax function is used to classify the question texts in teaching classrooms.

## 3. Results and Discussion

### 3.1. Comparison of Classification Results of Different Models of Teacher Questioning

CNN is classified according to the dimension of the question content. Assuming that there are 4500 questions to be classified, the content of the predicted questions is as follows: the basic knowledge point type is “0”, the question information type is “1”, the self-management type is “2”, and each question has 1500 questions. The confusion matrix at the end of the classification is shown in Table 2.

Over 80% of the question classifications are correct. The classification results of different models in the dimension of question content are shown in Figure 7.

In Figure 7, the overall performance of the CNN model is better than that of LSTM in the classification results of teacher's question content dimensions. The accuracy of CNN is higher. The classification accuracy rate of essential knowledge points is up to 86.3%. LSTM is only 79.2%. CNN is improved by 8.96%. The accuracy rate of the classification results of the three categories is small, but the CNN model is still better. In terms of recall rate and F1 value, the question classification results of the two models for basic knowledge points are better than the other two categories. The main reason lies in the unbalanced distribution of data volume during data sampling.

The classification results of different models in the question type dimension are shown in Figures 8 and 9.

In Figures 8 and 9, the overall performance of the CNN model is better than LSTM in the dimensional classification results of teacher question types. CNN has a higher accuracy rate. Prompt questions have the highest classification accuracy, reaching 87.82%. LSTM is only 83.2%. CNN is improved by 4.95%. This is because CNN can better obtain short text information. In terms of accuracy, the memorizing classification results are less effective than the other four types. Among them, the most accurate one is the suggestive question. The CNN model is the highest, reaching 99%. In terms of recall rate and F1 value, suggestive questions are less effective than the other four types of classification.

In Figure 10, the classification results of CNN in the question content classification dimension are compared with the performance of similar classification methods in literature [27] and literature [28]. In literature [27], it is studied whether experience can be used in the Knowledge Construction Phase (KCP) to change the type and function of teacher questions. The primary pedagogical goal of KCP revolves around the learner's demonstration of knowledge among learners with low language proficiency. Literature [28] studies a hypothetical mechanism: teacher perception. It is used to estimate the effect of kindergarten English learner status on teachers' perceptions of students' academic skills. The comparison results are shown in Figure 10.

In Figure 10, compared with the classification methods in other literature, the accuracy of CNN is higher, with an average of 85.7%. The performance is better.

Test results of the CNN network model on the training set and validation set are as follows.

The accuracy and loss value change curves of CNN models of different dimensions are shown in Figures 11 and 12.

Figures 11 and 12 are different classification methods for teacher question types. In the training process of the CNN model, the accuracy rate increases rapidly and then stabilizes. The loss value quickly shrinks and tends to stabilize. The training process performed well and could meet the requirements.

## 4. Conclusions

With the rapid development of AI, big data, and various network technologies, various industries are transforming toward intelligence. The traditional teaching model can no longer meet the requirements of information teaching. The reform of teaching mode is presented with new challenges through the analysis of AI-based smart classroom teaching mode and the application research of network technology in online classrooms. In the teaching process, teachers' classroom questioning is a part combined with computer technology. The intelligent analysis is carried out. A teacher's classroom questioning model based on deep learning is proposed. CNN-based and LSTM-based model classification methods are used to conduct classification experiments on teachers' classroom questions. CNN performed better. Some deficiencies still exist: the sample set of class question texts is small, and there are class imbalance problems. The accuracy of the model prediction still needs to be further improved. Future research will optimize the model and use a more complex neural network model for classification to improve the final classification effect.

## Figures and Tables

**Figure 1:** AI-based teaching model.

**Figure 2:** The talent training model of human-machine collaboration.

**Figure 3:** Forms of network technology teaching.

**Figure 4:** Intelligent analysis method of classroom questioning based on the deep learning algorithm.

**Figure 5:** CNN model composition structure.

**Figure 6:** LSTM network model composition structure.

**Figure 7:** Comparison of classification results between CNN and LSTM model.

**Figure 8:** CNN model classification results.

**Figure 9:** LSTM model classification results.

**Figure 10:** Comparison of CNN model classification results.

**Figure 11:** CNN model accuracy and Loss value change curve of the question content dimension.

**Figure 12:** CNN model accuracy and Loss value change curve of question type dimension.

**Table 1:** Distribution of the corpus of the simulated experimental data set.

Teacher question type	Dimension of the question content			Question type				
	Basic knowledge points	Topic information	Management type	Basic understanding and memory	Prompt	Analysis	Application class	Evaluation
Training set	903	1146	777	690	1353	852	438	234
Validation set	301	382	259	230	451	284	146	78
Test set	301	382	259	230	451	284	146	78
Total	1505	1910	1295	1150	2255	1420	730	390

**Table 2:** Confusion matrix for CNN classification.

	Predict the number of correct classifications			
	Teacher's question type	Basic knowledge	Subject information	Management type
The actual number of correct classifications	Basic knowledge	1295	57	83
	Subject information	178	1287	134
	Management type	27	156	1283

## Data Availability

The data used to support the findings of this study are available from the corresponding author upon request.
